# PCA-Based Incremental Extreme Learning Machine (PCA-IELM) for COVID-19 Patient Diagnosis Using Chest X-Ray Images

**DOI:** 10.1155/2022/9107430

**Published:** 2022-07-04

**Authors:** Vinod Kumar, Sougatamoy Biswas, Dharmendra Singh Rajput, Harshita Patel, Basant Tiwari

**Affiliations:** ^1^Koneru Lakshmaiah Education Foundation, Vaddeswaram, India; ^2^Vellore Institute of Technology, Vellore, India; ^3^Hawassa University, Awasa, Ethiopia

## Abstract

Novel coronavirus 2019 has created a pandemic and was first reported in December 2019. It has had very adverse consequences on people's daily life, healthcare, and the world's economy as well. According to the World Health Organization's most recent statistics, COVID-19 has become a worldwide pandemic, and the number of infected persons and fatalities growing at an alarming rate. It is highly required to have an effective system to early detect the COVID-19 patients to curb the further spreading of the virus from the affected person. Therefore, to early identify positive cases in patients and to support radiologists in the automatic diagnosis of COVID-19 from X-ray images, a novel method PCA-IELM is proposed based on principal component analysis (PCA) and incremental extreme learning machine. The suggested method's key addition is that it considers the benefits of PCA and the incremental extreme learning machine. Further, our strategy PCA-IELM reduces the input dimension by extracting the most important information from an image. Consequently, the technique can effectively increase the COVID-19 patient prediction performance. In addition to these, PCA-IELM has a faster training speed than a multi-layer neural network. The proposed approach was tested on a COVID-19 patient's chest X-ray image dataset. The experimental results indicate that the proposed approach PCA-IELM outperforms PCA-SVM and PCA-ELM in terms of accuracy (98.11%), precision (96.11%), recall (97.50%), F1-score (98.50%), etc., and training speed.

## 1. Introduction

The World Health Organization (WHO) identified COVID-19 (virus known as SARS-CoV-2) as a worldwide pandemic in February 2020. This triggered never expected counter-measures, such as the closure of cities, districts, and foreign travel. Coronaviruses (CoV) are death-defying viruses that may cause severe acute respiratory syndrome (SARS-CoV). Various researchers and institutions have attempted an effective solution from different possible diminutions in encountering the COVID-19 pandemic. Multimedia dataset (audio, picture, video, etc.) is booming in a massive amount of text information as civilization enters the information era. Image classification has become more essential as the need for real-world vision systems grows [1] and has recently attained a lot of attention from many researchers. It has evolved into one of the most essential operations, serving as a requirement for all other image processing operations. Image classification using learning algorithms is a special open issue in image processing that has sparked a lot of interest due to its promising applications. In general, an image categorization system has two primary processes. The first stage is to create an effective image representation that has enough information about the image to allow for classification further. The second step is to use a good classifier to classify the new image. Thus, there are two major challenges to consider when improving picture classification performance: dimensionality reduction and classifier. Apart from computer vision and image operation, one of the most important stages in image classification is feature extraction which determines the invariant characteristic of images when using computer devices to assess and deal with image data.

In a practical scenario, feature extraction has been applied in many fields like historic structures, medical image processing, remote image sensing, etc. The image's essential lower-level qualities include color, texture, and shape. The color feature has globality, which may be retrieved using tools such as the color histogram, color set, and color moment. It might simply explain the proportions of different colors across the image. The useful characteristic is color for identifying photos that are difficult to distinguish automatically, and the spatial variation should be ignored. However, it is unable to explain the image's local distribution as well as the description of the distinct colors' spatial positions. Image classification with feature extraction using incremental extreme learning machines is proposed in this paper. Firstly, on the COVID-19 dataset of chest X-ray images, features were extracted from an image using PCA. Eventually, the SVM, ELM, and IELM are applied to image classification [2] once the dimension is reduced by PCA method. Different metrics were employed to achieve the robust evaluation: classification accuracy, recall, precision, F-score, true-negative rate (TNR), true-positive rate (TPR), AUC, G-mean, precision-recall curve, and receiver operating characteristics (ROC) curve.

The paper is arranged in the following sequence: several related approaches have been discussed in Section 2. The suggested technique is described and critiqued in Section 3.  Section 4 contains a description of PCA and feature extraction techniques. Subsections 4.1–4.6 contain different algorithmic approaches that are compared with the proposed method. In Section 5, the proposed method and algorithm have been discussed.  Section 6 describes the different evaluation criteria that are used.  Section 7 discusses the experimental setup that has been used.  Section 8 describes the dataset. Finally, Section 9 discusses the experimental results, and the research is concluded.

## 2. Related Works

The content of image features comprises color, texture, and other visual elements. The extracted content from visual features is the main component for analyzing the image. In this segment, some of the earlier work based on PCA and other feature extraction techniques along with different classification techniques has been discussed.

Sun et al. [3] suggested an image classification system based on multi-view depth characteristics and principal component analysis. In this method, depth features are extracted from the image, and from RGB depth, characters are independently extracted and PCA is applied to reduce dimension. The Scene15 dataset, Caltech256 dataset, and MIT Indoor datasets are used in the evaluation process. Eventually, the SVM [4] is used to classify images. The method's performance is demonstrated by the experimental results.

Mustaqeem and Saqib [5] suggested a hybrid method that is based on PCA and SVM. PROMISE (KC1: 2109 observations, CM1: 344 observations) data from NASA's directory have been used for the experiment. The dataset was divided into two parts: training (KC1: 1476 observations, CM1: 240 observations) and testing (KC1: 633 observations, CM1: 104 observations). Principal components of the features are extracted by PCA, and it helps in dimensionality reduction and minimizing time complexity.

In addition to this, SVM is used for further classification, and for hyperparameter tuning, GridSearchCV is used. From this, precision, recall, F-measure, and accuracy for KC1 dataset analysis are 86.8%, 99.6%, 92.8%, and 86.6%, respectively, and for CM1 dataset analysis, precision, recall, F-measure, and accuracy are 96.1%, 99.0%, 97.5%, and 95.2%, respectively. Similarly, Castaño et al. [6] provide a deterministic approach for starting ELM training based on hidden node parameters with activation function. The hidden node parameters are calculated with the help of Moore–Penrose generalized inverse, whereas the output node parameters are recovered through principal component analysis. Experimental validation with fifteen well-known datasets was used to validate the algorithm. The Bonferroni–Dunn, Nemenyi, and Friedman tests were used to compare the results obtained. In comparison with later ELM advancements, this technique significantly reduces computing costs and outperforms them.

Mateen et al. [7] suggested VGG-19 DNN-based DR model with better performance than AlexNet and the spatial invariant feature transform (SIFT) in terms of classification accuracy and processing time. For FC7-SVD, FC7-PCA, FC8-SVD, and FC8-PCA, respectively, classification accuracies are 98.34%, 92.2%, 98.13%, and 97.96% by using SVD and PCA feature selection with fully connected layers.

Zhao et al. [8] suggested extreme learning machines with no iteration along with supervised samples are used for model building as a class incremental extreme learning machine. The algorithm is shown to be stable and has almost equivalent accuracy of batch learning. Similarly, Huang and Chen [9] proposed an algorithm that analytically calculates hidden nodes' output after randomly producing and adding computational nodes to the hidden layer as a convex incremental extreme learning machine. Using a convex optimization, the existing hidden node output is calculated again. This can converge faster while maintaining efficiency and simplicity.

Zhu et al. [10] proposed a principal component analysis (PCA)-based categorization system with kernel-based extreme learning machine (KELM). Based on the resultant output, this model achieves better accuracy than SVM and other traditional classification methods. For the classification of HSIs, Kang et al. [11] developed the PCA-EPF extraction approach. In this research work, they have proposed the combination of PCA and standard edge preserving filtering (EPF)-based feature extraction. The proposed method achieves better classification accuracy with limited training samples. Similarly, Perales-González et al. [12] introduced a new ELM architecture based on the negative correlation learning framework dubbed negative correlation hidden layer ELM (NCHL-ELM). This model shows better accuracy when compared with other classifications by integrating a parameter into each node in the original ELM hidden layer.

Based on fractal dimension technology, Li et al. [13] suggested an enhanced ELM algorithm (F-ELM). By reducing the dimension of the hidden layer, the model improves in training speed. From the experimental results, it can be concluded that as compared to the standard ELM technique, the suggested algorithm significantly reduces computing time while also improving inversion accuracy and algorithm stability.

Because of the complexity of the data models, deep learning is incredibly pricey to train. Furthermore, deep learning necessitates the use of high-priced GPUs and hundreds of computer machines. There is no simple rule that can help you choose the best deep learning tools since it necessitates the understanding of topology, training technique, and other characteristics, whereas the simple ELM is a one-shot computation with a rapid learning pace. But the biggest advantage in IELM is the ability to randomly increase hidden nodes incrementally and analytically fix the output weights. The output error of the IELM rapidly diminishes as the number of hidden neurons increases.

In our method, SVM, ELM, and IELM based on the PCA technique are employed for image classification [14] for COVID-19 patient detection using the COVID-19 chest X-ray dataset. A summary of the most recent and related research works is described in Table 1 [3, 5–13].

## 3. Proposed Methodology

The back propagation (BP) approach is commonly used to train multi-layer perceptron (MLP). Various algorithms can be used to train this typical architecture. Gradients and heuristics are two types of algorithms that are commonly used. These algorithms have a few things in common: they have a hard time dealing with enormous amounts of data, and they have a slow convergence rate in these situations. Huang et al. (Huang et al.) [15] introduced the extreme learning machine as a solution to this problem.

The typical computing time required to train an SLFN using gradient-based techniques is reduced by this algorithm. The ELM, on the other hand, has several flaws. The randomly generated input weights and bias for ELM [16] result in some network instability. In case if there are outliners in the training data, then the hidden layer's output matrix will have ill-conditioned problems and it results in low generalization performance and lower forecasting accuracy. There are two types of ELM called fixed ELM and IELM [17]. In comparison with the ELM, the output error of the IELM rapidly diminishes and it tends toward zero with the growth in number of hidden neurons (Huang et al.) [15]. In online continuous learning regression and classification problem, this approach is very prominent (Xu and Wang; Zhang et al.) [18, 19].

A trained classifier can be obtained after training the classifiers with a sufficient amount of image data and then fed into the trained classifier for observation and analysis.

## 4. Feature Extraction

A single feature cannot describe the image feature and quality properly. The image classification will not yield acceptable results unless distinguishing features are described. Three images corresponding to three viewpoints are placed on each RGB color image. Our method uses PCA to extract the image's important information and minimize the input dimension [20–23].

### 4.1. Classification of Images and PCA Feature Extraction

Extracting useful features from an image is a prominent task in image classification, and principal component analysis (PCA) is used for this purpose. PCA uses orthogonal transformation and converts variables to fewer independent components than the original variables. The output data with this approach will not lose important data features, and PCA loadings can be used for the identification of important data. A multivariate statistical analysis approach is used by PCA, which can perform linear transformation of numerous variables to pick a few key variables. PCA transforms data using eigenvectors from N-dimension to M-dimension where *M* < *N*. The new features are a linear mixture of the old ones, allowing them to capture the data's intrinsic unpredictability with little information loss.  Figure 1 reveals the steps of the proposed model.

Suppose that the research object has *p* indexes, these indexes are regarded as *p* random variables and represented as *X*_1_, *X*_2_, , *X*_*p*_. With this, new indexes are created by combining *p* random variable *F*_1_, *F*_2_, ..., *F*_*p*_, which can mirror the data from the original indexes [24]. The independent replacement indexes reflect the original indexes' essential information.

(1) $$\begin{array}{c} F_{1}=a_{11}X_{1}+a_{12}X_{2}+\cdots +a_{1p}X_{p},\\ F_{2}=a_{21}X_{1}+a_{22}X_{2}+\cdots +a_{2p}X_{p},\\ \ldots \ldots \ldots ,\\ F_{p}=a_{p1}X_{1}+a_{p2}X_{2}+\cdots +a_{pp}X_{p}. \end{array}$$

The following are the PCA stages in detail:

(1) *Data standardization*: The following calculation formula is used to standardize the matrix *X*:
  (2) $$\begin{array}{c} y_{\text{ij}}=\frac{x_{\text{ij}}-{\bar{x}}_{j}}{\sqrt{\text{Var}\left(x_{j}\right)}}, \end{array}$$
where *X* = {*x*_*ij*_}, *Y* = {*y*_*ij*_}, where *i* = 1, 2, ..., *n* and *j* = 1, 2, ..., *p*,
  (3) $$\begin{array}{c} \bar{x}=\frac{1}{n}\sum_{i=1}^{n}x_{\text{ij}},\\ \mathrm{var}\left(\text{xj}\right)=\frac{1}{n-1}\sum_{i=1}^{n}{\left(x_{\ddot{\text{ij}}}-{\bar{x}}_{j}\right)}^{2}. \end{array}$$
(2) The following formula is used to solve the correlation coefficient matrix *R*:
  (4) $$\begin{array}{c} R=\frac{Y^{T}Y}{n-1}. \end{array}$$
(3) The following formula is used to calculate the eigenvalue and eigenvector of the coefficient matrix:
  (5) $$\begin{array}{c} \left|R-\lambda I_{P}\right|=0. \end{array}$$
The calculated eigenvector is *a*_*i*_ = (*a*_*i*1_, *a*_*i*2_, ... , *a*_*ip*_), where *i* = 1, 2, 3, 4,…………., *p*, and the eigenvalue is *λi* (*i* = 1, 2, ..., *p*). To get a collection of main components Fi, the eigenvalues are sorted in descending order:
  (6) $$\begin{array}{c} F_{i}=a_{i1}Y_{1}+a_{i2}Y_{2}+\cdots +a_{ip}Y_{p}. \end{array}$$
(4) The following are the main factors to consider kth primary component contribution rate and expressed as
  (7) $$\begin{array}{c} \lambda_{k}{\left(\sum_{j=1}^{P}\lambda_{j}\right)}^{-1}. \end{array}$$

The rate of the first *k* primary components' cumulative contribution is expressed as

(8) $$\begin{array}{c} \sum_{j=1}^{k}\lambda_{j}{\left(\sum_{j=1}^{P}\lambda_{j}\right)}^{-1}. \end{array}$$

The first principal component, *F*_1_, is the one with the highest variance out of all the combinations of *Y*_1_, *Y*_2_, ..., *Y*_*p*_; the second principal component *F*_2_ is one with the highest variance among all the combinations of *Y*_1_, *Y*_2_, ..., *Y*_*p*_, and they have no relation with *F*_1_.

### 4.2. SVM

Several algorithms have been implemented and suggested in machine learning to solve the classification problem. Among the different classification problems, support vector machine (SVM) is one of the supervised algorithms in machine learning with [5, 25] the advantages as follows:

- It employs L2 regularization to overcome overfitting problems.
- Even with minimal data, provide suitable findings.
- Different kernel functions to match the features' complicated functions and interactions.
- Manages the data nonlinearity.
- The model is stable thanks to the hyper-plane splitting rule.
- Analyzes the data with a high degree of dimensionality.

Instead of focusing on decreasing prediction error, SVM focuses more on optimizing classification decision boundaries, which is why the hyper-plane is used to separate classes. If the data dimension is *n* and the hyper-plane is a (*n* − 1) vector function, then it can be represented mathematically as follows:

(9) $$\begin{array}{c} y=w_{0}x_{0}+w_{1}x_{1}+\cdots +w_{n-1}x_{n-1}+b. \end{array}$$

It also signifies, in a broader sense,

(10) $$\begin{array}{c} y=w^{T}x+b, \end{array}$$

where *x* denotes the input feature vector, *w* is the weight vector, and *b* is the bias. By adjusting *w* and *b*, several hyper-planes can be created, but the hyper-plane with the best margin will be chosen. The largest feasible perpendicular distance between each class and the hyper-plane is defined as ideal margin. The cost function or objective function is minimized to get the best margin. The cost function may be written as follows:

(11) $$\begin{array}{c} J\left(w\right)=\frac{1}{2}\left\|w^{2}\right\|+\frac{1}{n}\sum_{i=0}^{n}\text{max}\left(0,\left(1-y_{i}*\left(w^{T}x+b\right)\right)\right., \end{array}$$

Even if the predictions are right and the data are correctly categorized by hypothesis, SMV utilized to penalize any *y*_*i*_ that are close to the borders (0 < *y*_*i*_ < 1). The main goal is to figure out optimal *w* value to minimize *J*(*w*), so differentiating Eq. 11 concerning *w*, we get the gradient of a cost function as follows:

(12) $$\begin{array}{c} \nabla_{w}J\left(w\right)=\frac{\partial J\left(w\right)}{\partial w},\\ =\frac{1}{n}\sum_{i=0}^{n}\left\{\begin{array}{cc} w, & \text{if max}\left(0,\right.\left(1-y_{i}*\left(w^{T}x+b\right)\right),\\ w-y_{i}x_{i\;}, & \text{otherwise}. \end{array}\right.. \end{array}$$

As far as we have calculated ∇_*w*_*J*(*w*), weights of *w* can be updated as

(13) $$\begin{array}{c} W_{\text{new}}=W_{\text{old}}-\alpha \left[J\left(w\right)\right]. \end{array}$$

We go through the procedure again and again until smallest *J*(*w*) discovered. Because data are rarely linearly separable, we must sketch a decision boundary between the classes rather than using a hyper-plane to separate them. We will need to convert (13) into a decision boundary to deal with the dataset's nonlinearity:

(14) $$\begin{array}{c} y=w\cdot \phi \left(x\right)+b. \end{array}$$

*ϕ*(*x*)  is the kernel function in (14). There are various types of kernel functions that may be used to create SVM, such as linear, polynomial, and exponential, but we will use the radial basis function in this model (RBF). Distance parameter that is used is Euclidean distance, and the smoothness of the borders is defined by the parameter *σ*.

(15) $$\begin{array}{c} \phi \left(x\right)=\exp\left(-\frac{x-{\bar{x}}^{2}}{2\sigma^{2}}\right), \end{array}$$

where $x-{\bar{x}}^{2}$ is the square of Euclidean distance between any single observation *x* and mean of the training sample *x*.

### 4.3. PCA-SVM

The motive of the support vector machine (SVM) [3] is to find the best possible hyper-plane that will separate two planes on the training set. The coefficient of the hyper-plane is *w* that we have to project. It uses structural risk minimization theory to build the best hyper-plane segmentation in the feature space and a learning editor to achieve global optimization.

Assume the training data, (*x*_1_, *y*_1_), (*x*_2_, *y*_2_),…, (*x*_*n*_, *y*_*n*_) ∈ *R*^*n*^, *y* ∈ {−1,1}.

This could be projected into a hyper-plane:

(16) $$\begin{array}{c} \left(\omega \cdot x\right)+b=0,\omega \in R^{n}b\in R. \end{array}$$

For the normalization,

(17) $$\begin{array}{c} y_{i}\left(\omega \cdot x_{i}\right)+b\geq 1,\;i=1,2,\ldots ,l. \end{array}$$

The classification of the interval is equal to 2/*ω*, when the maximum interval is equal to the minimum *ω*^2^.

Before classifying the data through SVM, the necessary features from the image data need to be extracted. The high-dimensional data can be converted to the low-dimensional data with this approach. For this, the PCA method as a feature extraction through convergence matrix and eigenvalue proportion calculation is used. PCA-based SVM is the method that is used for classification and regression. After that, SVM is used to classify low-dimensional data.  Figure 2 depicts the working flow of PCA-SVM. Once the parameter optimization is done, the model is ready to predict categorization.

### 4.4. Extreme Learning Machine (ELM)

An extreme learning machine is a single hidden layer feedforward network that can be used for both classification and regression. In ELM [26], weights between the input layer, hidden layer, and biases are randomly generated. The output weights are calculated using the generalized Moore–Penrose pseudo-inverse. ELM performs faster than other feedforward networks [27] and outperforms other iterative methods.  Figure 3 shows the basic network architecture of ELM.

Suppose [**x**_**i**_, **t**_**i**_] denotes *N* training samples, wherein training instances *iϵ* 1, 2, 3,…………, *N* and **x**_**i**_ = [*x*_*i*1_, *x*_*i*2_,…, *x*_*im*_]*T ϵ R*^*m*^ denotes *i*^th^ training instance and its desired output **t**_**i**_ = [*t*_*i*1_, *t*_*i*2_,…, *t*_*iC*_ ]^*T*^*ϵ R*^*C*^.

Let the number of input features and number of neurons be equal and represented by *m*; similarly, let *L* be the number of hidden neurons. The number of output neurons and number of classes are equal and denoted by *c*.  Figure 4 [24] shows the flowchart of the principal component analysis [28]. The input weight matrix is represented by **U** = [**u**_**1**_, **u**_**2**_,…, **u**_**j**_,…**u**_**L**_]^*T*^∈*R*_*L*×*m*_, and the hidden neuron bias is represented by **b** = [*b*_1_, *b*_2_,…, *b*_*j*_,…*b*_*L*_]^*T*^∈*RL*. **u**_**j**_ = [*u*_*j*1_, *u*_*j*2_,…*u*_*jm*_] are the connecting weights between the *j*^th^ hidden neuron with the input neurons. Bias of the *j*^th^ hidden neuron is *bj*, and *j*th hidden layer output for *i*^th^ instance is represented by

(18) $$\begin{array}{c} h_{ij}=g\left(u_{j}x_{i}+b_{j}\right). \end{array}$$

Here, activation function is represented by *g*. For all the training instances hidden layer output is represented by **H** and can be represented by

(19) $$\begin{array}{c} H\;=\left(\begin{array}{ccc} h_{11} & h_{12} & h_{1L}\\ \ldots & \ldots & \ldots \\ h_{j1} & h_{j2} & h_{jL}\\ \ldots & \ldots & \ldots \\ h_{N1} & h_{N2} & h_{NL} \end{array}\right). \end{array}$$

Between the hidden layer and the output layer, the output weight ***β*** can be computed using Eq. (20). Linear activation function is used by the output layer in this computation.

(20) $$\begin{array}{c} \beta =H^{†}T. \end{array}$$

Here,

(21) $$\begin{array}{c} \beta ={\left[\beta_{1}^{T},\ldots ,\beta_{j}^{T},\ldots ,\beta_{L}^{T}\right]}_{L\times C}^{T}. \end{array}$$

The vector ***β***_***j***_ = [*β*_*j*1_,…, *β*_*jk*_,…, *β*_*jC*_]^*T*^, where *j* = (1, 2, 3,…..…, *L*) represents the connecting weights between the *j*^th^ hidden neuron and the *k*^th^ output neuron. The predicted outcome of all the output neurons for all training instances is represented as

(22) $$\begin{array}{c} f\left(x\right)=\;H\beta . \end{array}$$

Here, the output function is **f**(**x**) = [*f*_*k*_(**x**),…, *f*_*C*_(**x**)]. From Eq. 23, label for class **x** can be predicted.

(23) $$\begin{array}{c} \text{label}\left(x\right)=\arg\max f_{k}\left(x\right),\;k=1,\ldots ,C. \end{array}$$

### 4.5. PCA-ELM : Classification Method Based on PCA-ELM

In the PCA technique [6], variables are first scaled. The different steps of PCA that has been applied in PCA-ELM are

1. Scaling of trained data.
2. Covariance matrix evaluation.
3. Eigenvalues for the covariance matrix along with eigenvectors are defined.
4. Evaluating the principal components.

The output from PCA is given as an input to ELM [29]. The process of PCA-ELM [30] is shown in Figure 5.

### 4.6. ELM

Compared to the other neural networks, the ELM learns faster as there is no need to adjust hidden nodes and provides better generalization capability. But there are various flaws with the ELM. Randomly generated bias and input weights in ELM network [31] are results in some network instability. Training data outliers from the hidden layer's output matrix result in poor network generalization performance. In comparison to the ELM, the output error of the IELM rapidly diminishes and resolves the issue of very small weights of output and validity of hidden layer neurons. In online continuous learning, it is appropriate for regression and classification tasks.

The IELM [32] network model structure is shown in Figure 6. Suppose the size of input, hidden nodes, and outputs are *m*, *l*, and *n*, respectively, and *ω*_*i*_ is the input weight matrix with *l* × *m*  dimension of the current hidden layer neuron and uniformly distributed between random numbers [−1,  1]. The bias of the ith hidden node *b*_*i*_ is a random number between [−1,  1] uniformly distributed, the activation function for the hidden layer neuron is sigmoid function given by (24), and output weight matrix *β* is with *l* × *n* dimension.

The hidden node activation function (sigmoid) is given by

(24) $$\begin{array}{c} g\left(x\right)=\frac{1}{1+e^{-x}}, \end{array}$$

where *x* is the input matrix.

A matrix *X* is of *m* × *N* dimension, and it represents *N* dataset input. *Y* is a *n* × *N* matrix that represents the output where *N* datasets for a training set {(*X*, *Y*)}. Training steps of IELM algorithm are described as follows:

**Step 1 .**

In the initialization phase, suppose *l*  = 0 and *L* is the maximum number of the hidden nodes. Output *Y* is defined in terms of the initial value of the residuals *E* (difference between target and actual error) is set to be the and *ε* is the expected training accuracy.

**Step 2 .**

Training phase, while *l* < *L* and *E* > *ε*

(1) Hidden nodes *l* will be increased by 1, i.e.,
  (25) $$\begin{array}{c} l=l+1. \end{array}$$
(2) Hidden layer neuron *O*_*l*_ is evaluated randomly from input weights *ω*_*l*_ and bias *b*_*l*_.
(3) Output of the activation function *g*(*x*′) is calculated for the node *O*_*l*_ (*b*_*l*_ needs to be extended into a *l* × *N*  vector *b*_*l*_).
  (26) $$\begin{array}{c} x^{\prime }=\omega_{l}x+b_{l}. \end{array}$$
(4) Hidden layer neuron output vector $\bar{H}$ can be calculated from
  (27) $$\begin{array}{c} \bar{H}=g\left(x^{\prime }\right). \end{array}$$
(5) Output weight for *O*_*l*_ can be evaluated from
  (28) $$\begin{array}{c} \bar{\beta }=\frac{E\cdot {\left(\bar{H}\right)}^{T}}{\bar{H}\cdot {\left(\bar{H}\right)}^{T}}. \end{array}$$
(6) After increasing the new hidden node, residual error is calculated:
  (29) $$\begin{array}{c} E^{\prime }=E-\bar{\beta }\bar{H}. \end{array}$$

The network error rate can be reduced by the output weight *O*_*l*_. All these steps will iteratively work till the residual error becomes smaller than *ε*. The training process restarts through the determination of the random input weight *ω*_*l*_ and the bias *b*_*l*_. Whether the trained network has fulfilled the desirable result or not can be determined from {(*X*′, *Y*′)} set.

## 5. Proposed PCA-Based Incremental ELM (PCA-IELM)

An orthogonal transformation is used to extract meaningful characteristics from data in PCA [33]. PCA may also be used to minimize the dimensions of a large data collection. Principal components from COVID-19 X-ray images are extracted using PCA and given as input to IELM which gradually adds concealed nodes produced at random. A conventional SLFNs function with *n* hidden nodes can be expressed as

(30) $$\begin{array}{c} f_{n}\left(x\right)=\sum_{i=1}^{n}\beta_{i}g_{i}\left(x\right),\;x\in R^{\text{d}},\beta_{i}\in R. \end{array}$$

where  *g*_*i*_(*x*)=*g*(*a*_*i*_, *b*_*i*_, *x*) denotes the output of the ith hidden node:*g*_*i*_(*x*)=*g*(*a*_*i*_.*x*+*b*_*i*_) (for additive nodes) or *g*_*i*_(*x*)=*g*(*b*_*i*_*x* − *a*_*i*_).

The ith hidden layer and the output node are linked with output weights *β*_*i*_. Hidden nodes are randomly added to the existing networks in IELM. The randomly generated hidden node parameters *a*_*i*_ and *b*_*i*_ and fixed output weight are *β*_*i*_.

Suppose the residual error function for the current network *f*_*n*_ is defined as *e*_*n*_≅*f* − *f*_*n*_ . where *n* is the number of hidden nodes and *f* ∈ *L*^2^(*x*)  is the target function. IELM is mathematically represented as

(31) $$\begin{array}{c} f_{n}\left(x\right)=f_{n-1}\left(x\right)+\beta_{n}g_{n}\left(x\right). \end{array}$$

## 6. Evaluation Criteria for Effective Measure of Model

For evaluation of the different models, generally, the confusion matrix is prepared.  Table 2 defines a simple representation of the confusion matrix [34, 35], and it can classify between predicted and actual values. From the confusion matrix, we can derive different performance metrics, e.g., accuracy, precision, recall, sensitivity, and F-score. To assess the model, nine different metrics are calculated by formula as given in Table 3 [36].

## 7. Experimental Setup

The whole experiment was performed on a system having a configuration of 10th Generation Intel (*R*) Core (TM) i7-10750H CPU @ 2.60 GHz processor, 8 GB RAM, and NVIDIA GTX graphics 1650TI. The code is written in *Python* 3.10.0 and uses Jupyter Notebook as a debugger, which can be installed from the link: https://jupyter.org/install.

## 8. Dataset Description

The COVID-19 chest X-ray images [37] dataset encompasses a total of 13808 images in which 3616 COVID-19 positive cases (26.2%) along with 10,192 (73.8%) normal cases are downloaded from Kaggle. COVID-19 and normal patient chest X-ray images are kept in separate files. Dataset was divided into training and testing images which had been done randomly with a condition that testing images will not be repeated in training images. During the experiment, 80% of the total images were used for training and 20% for testing. All images have the same dimension (299 × 299) pixels in the PNG file format.  Figure 7 demonstrates the X-ray images of normal and COVID-19 cases.

The histogram of an image gives a global description of the image's appearance. It represents the relative frequency of occurrences of various intensity values in an image. In the histogram of the COVID-19 image, the intensity value is highest between bins 14–15, whereas in the normal image the histogram has the highest intensity value at bins 16–17. This difference in the color intensity value assists in making the distinction between COVID-19 and normal images.  Figure 8 demonstrates the histogram plot of normal and COVID-19 images.  Figure 9 shows the training images for X-ray images of COVID-19 and normal.

Because PCA uses orthogonal transformation to convert all features into a few independent features, all features are considered during the feature selection process. The data to be processed are reduced to a set of features called a “reduced representation set.”

## 9. Results and Discussion

In this segment, we present the outcomes and analysis of the experiments performed in the COVID-19 patient prediction using the chest X-ray dataset. From the experimental results, the proposed method shows better performance in terms of accuracy, precision, recall, F1-score, AUC, G-mean, and other parameters. For each model, PCA-SVM, PCA-ELM, and PCA-IELM, a separate confusion matrix is formed. All the performance metrics values are derived from the confusion matrix (Tables 4–6). Classification accuracy gained by the proposed method PCA-IELM is 98.11% over the chest X-ray dataset, which suggests better results than the other two models, PCA-based SVM (91.8%) and PCA-based ELM (93.80%) in terms of accuracy. Sometimes, performance metrics' accuracy may be misleading and can misclassify instances. So, other metrics are also taken into consideration to confirm the claim made by the classifier. PCA-IELM has the highest precision value of 96.11%. That means PCA-IELM is 96.11% reliable in making decisions, whereas models PCA-SVM and PCA-ELM record less precision, 84.3% and 88.3%, respectively. Similarly, for the proposed method PCA-IELM, other metrics (refer to Figure 10) recall, *F*_1_-score, TPR, TNR, and G-mean are considerably higher than the other two methods, PCA-SVM and PCA-ELM.

The geometric mean (G-mean) is a statistic that analyzes categorization performance across majority and minority classes. Even if negative examples are correctly labelled as such, a poor G-mean suggests weak performance in identifying positive occurrences. This statistic is essential for preventing overfitting the negative class while underfitting the positive class, since the COVID-19 dataset understudy is also class imbalanced (IR = 2.81). Even then, the PCA-ELM model indicates good performance by attaining the highest G-mean value of 98%. Similarly, PCA-SVM and PCA-ELM have 88% and 90.5% success rates, respectively.

Table 7 demonstrates the performance variation (sensitivity, specificity, precision, F1-score, accuracy) based on different counts of hidden nodes in the range of 10–150 with an interval of 10 hidden nodes. Training and testing accuracies of PCA-IELM demonstrated almost the same behavior on the COVID-19 dataset (refer to Figure 11). There is moderate variation in the accuracy of PCA-IELM with respect to different numbers of hidden nodes. The accuracy at 10 numbers of hidden nodes was found to be 97.73%, and 98.11% was achieved at 140 numbers of hidden nodes in the PCA-IELM model and beyond (refer to Table 7).

When there is a moderate to large class imbalance, precision-recall curves should be drawn. Here, the COVID-19 dataset is imbalanced with an imbalance ratio (IR) of 2.81. It is worth noticing that precision is also called the positive predictive value (PPV). Moreover, recall is also known as sensitivity, hit rate, or true-positive rate (TPR). It means they talk about positive cases and not negative ones. Most machine learning algorithms often involve a trade-off between recall and precision. A good PR curve has a greater AUC (area under curve). Figures 12(b), 13(b), and 14(b) depict PR curves.  Figure 13(b) shows the greater AUC, which is an indication of the better performance of PCA-IELM than the other two models. In addition to these, ROC of Figure 14(a) also grabs more AUC than two other Figures 12(a) and 13(a). Therefore, PCA-IELM claims better performance than PCA-SVM and PCA-IELM. The proposed PCA-IELM model outperforms other previously developed models for identification of COVID-19 patients from chest X-ray image (refer Table 8 [38–47]). As far as the training and testing time taken by the proposed model PCA-IELM is concerned, it was higher (refer to Table 9) because the execution of the model happened in an incremental way and not in one go.

## 10. Conclusions

In this paper, an effective classification model is proposed on the COVID-19 chest X-ray image dataset using principal component analysis (PCA) and incremental extreme learning machine (IELM). This study established the valuable application of the ELM model to classify COVID-19 patients from X-ray images by developing the PCA-IELM model. The proposed PCA-based IELM algorithm is an efficient IELM-based algorithm. The hidden node parameters are measured by the information returned to the PCA in the training dataset, and using the Moore–Penrose generalized inverse output, the node parameters are determined. PCA-IELM utilizes the best feature of IELM, which is to increase hidden nodes incrementally and wisely determine the output weights, whereas ELM requires you to set the appropriate number of hidden nodes manually, and this is similar to the hit and trial method. In comparison with the ELM, the output error of the IELM rapidly reduces and is near to zero as the number of hidden neurons increases. It was observed that as the number of hidden nodes increased, the performance of the PCA-IELM increased and it became stable at 150 hidden nodes. PCA-IELM outperforms PCA-SVM and PCA-ELM in terms of accuracy (98.11%), precision (96.11%), recall (97.50%), F1-score (98.50%), G-mean (98%), etc. The suggested research contributes to the prospect of a low-cost, quick, and automated diagnosis of the COVID-19 patient, and it may be used in clinical scenarios. This effective system can provide early detection of COVID-19 patients. As a result, it is helpful in controlling the further spread of the virus from an affected person. This is an intelligent assistance for radiologists to accurately diagnose COVID-19 in X-ray images.

## Figures and Tables

**Figure 1:** Flowchart of the proposed model (PCA-IELM).

**Figure 2:** Flowchart of PCA-SVM.

**Figure 3:** Network architecture of ELM.

**Figure 4:** Flowchart of the principal component analysis [24].

**Figure 5:** Process of PCA-ELM.

**Figure 6:** The structure of IELM.

**Figure 7:** Chest X-ray images of COVID-19 and normal.

**Figure 8:** Histogram for X-ray images of COVID-19 and normal.

**Figure 9:** Training images for X-ray images of COVID-19 and normal.

**Figure 10:** Performance comparison of different classifiers.

**Figure 11:** Accuracy variation with number of hidden nodes for PCA-IELM.

**Figure 12:** (a) Analysis of ROC curve and (b) analysis of precision-recall for PCA-SVM.

**Figure 13:** (a) Analysis of ROC curve and (b) analysis of precision-recall for PCA-ELM.

**Figure 14:** (a) Analysis of ROC curve and (b) analysis of precision-recall for PCA-incremental ELM.

**Algorithm 1:** SVM algorithm.

**Algorithm 2:** PCA-SVM algorithm.

**Algorithm 3:** ELM algorithm.

**Algorithm 4:** PCA-ELM algorithm.

**Algorithm 5:** IELM algorithm.

**Algorithm 6:** PCA-IELM algorithm.

**Table 1:** Similar work summarization.

SN	References	Applied method	Problem approached	Resulted outcome	Impediments
1	Sun et al. [3]	PCA of multi-view deep representation	Image classification	Comparison result from different databases	Limited classifiers are compared
2	Mustaqeem and Saqib [5]	Principal component-based support vector machine	Software defect detection	Better accuracy than other methods	No probabilistic explanation for SVM classification
3	Castaño et al. [6]	Pruned ELM approach based on principal component analysis	Classification	ELM model based on PCA	Limited classifiers are compared
4	Mateen et al. [7]	VGG-19 architecture with SVD and PCA	Fundus image classification	Better accuracy than other methods	Limited to nonimbalance data
5	Zhao et al. [8]	IELM	Activity recognition	Stable and similar accuracy to the batch learning method	Limited to batch learning
6	Huang et al. [9]	Convex incremental extreme learning machine	Convergence rate of IELM	Faster convergence rate	Limited classifiers are compared
7	Zhu et al. [10]	PCA and kernel-based ELM	Side-scan sonar image classification	Better classification accuracy with stable model	Classify underwater targets only
8	Kang et al. [11]	PCA-based edge-preserving features (EPF)	Hyperspectral image classification	Better accuracy than SVM	Parameters of EPFs are given manually
9	Perales-González et al. [12]	Negative correlation hidden layer for the ELM	Regression and classification	Better accuracy	Variety in the transformed feature space
10	Li et al. [13]	Improved ELM	Transient electromagnetic nonlinear inversion	Improves the inversion accuracy and stability	Less implementation in other industrial domains

**Table 2:** Confusion matrix.

Predicted			Total
Actual	TP (true positive)	FP (false positive)	TP + FP
	FN (false negative)	TN (true negative)	FN + TN
Total	TP + FN	TN + FP	ALL

**Table 3:** Performance evaluation measures [36].

SL	Measures	Formula
1.	Accuracy	TP+TN/TP+FP+TN+FN
2.	Specificity (TN_rate_)	TN/TN+FP
3.	FN_rate_	FN/TP+FN
4.	Sensitivity (TP_rate_)/recall	TP/TP+FN
5.	FP_rate_	FP/TN+FP
6.	Precision	TP/TP+FP
7.	G-mean	$\sqrt{{\text{ TP}}_{\text{rate}}\times {\text{TN}}_{\text{rate}}}$
8.	AUC	1+TP_rate_ − FP_rate_/2
9.	*F*_1_-score	2*∗*TP/2*∗*TP+FP+FN

**Table 4:** Confusion matrix for PCA-SVM.

Predicted			Total
Actual	819	152	971
	187	2985	3172
Total	1006	3137	4143

**Table 5:** Confusion matrix for PCA-ELM.

Predicted			Total
Actual	828	110	938
	147	3058	3205
Total	975	3168	4143

**Table 6:** Confusion matrix for PCA-IELM.

Predicted			Total
Actual	1192	48	1240
	30	2873	2903
Total	1222	2921	4143

**Table 7:** Performance variation based on different hidden nodes.

Number of hidden nodes	Performance metrics (%)				
	Sensitivity	Specificity	Precision	*F*_1_-score	Accuracy
10	94.13	96.23	93.74	95.19	97.73
20	94.16	96.19	93.36	95.19	97.73
30	94.24	96.35	94.48	95.24	97.74
40	93.98	96.07	93.01	94.98	97.70
50	94.11	96.16	93.09	95.11	97.71
60	94.18	96.28	93.45	95.18	97.73
70	94.73	96.82	94.69	95.64	97.75
80	94.84	96.79	94.86	95.29	97.75
90	94.25	96.77	94.92	95.36	97.75
100	94.03	96.11	93.11	95.02	97.71
110	94.17	96.24	93.22	95.16	97.73
120	94.48	96.46	94.59	95.71	97.75
130	94.10	96.15	93.19	95.11	97.71
140	97.62	98.12	96.33	96.50	98.11
150	97.54	98.35	96.12	96.83	98.11

**Table 8:** Proposed method and other related models' comparative analysis [38].

S.No.	Study	Method used	Number of cases	Type of images	Accuracy (%)
1	Ioannis et al. [39]	VGG-19	700 pneumonia, 504 healthy, 224 COVID-19 (positive)	Chest X-ray	93.48
2	Gunraj, Wang, and Wong [40]	COVID-Net	5526 COVID-19 (negative), 8066 healthy, 53 COVID-19 (positive)	Chest X-ray	92.4
3	Sethy et al. [41]	ResNet50þ SVM	25 COVID-19 (negative), 25 COVID-19 (positive)	Chest X-ray	95.38
4	Hemdan et al. [42]	COVIDX-Net	25 normal, 25 COVID-19 (positive)	Chest X-ray	90.0
5	Narin et al. [43]	Deep CNN ResNet-50	50 COVID-19 (negative), 50 COVID-19 (positive)	Chest X-ray	98
6	Ying et al. [44]	DRE-Net	708 healthy, 777 COVID-19 (positive)	Chest CT	86
7	Wang et al. [45]	M-Inception	258 COVID-19 (negative), 195 COVID-19 (positive)	Chest CT	82.9
8	Zheng et al. [46]	UNetþ3D deep network	229 COVID-19 (negative), 313 COVID-19 (positive)	Chest CT	90.8
9	Xu et al. [47]	ResNetþ location attention	175 healthy, 224 viral pneumonia, 219 COVID-19 (positive)	Chest CT	86.7
10	Tulin et al. [38]	DarkCovidNet	500 Pneumonia, 500 no-findings, 125 COVID-19 (positive	Chest X-ray	98.08
11	Proposed model	PCA-IELM	10,192 normal, 3616 COVID-19 (positive)	Chest X-ray	98.11

**Table 9:** Time elapsed during training and testing of models.

Dataset	Algorithm	Training time (s)	Testing time (s)
COVID-19 chest X-ray	PCA-SVM	0.027	0.022
	PCA-ELM	0.053	0.049
	PCA-IELM	12.353	9.525

## Data Availability

The data used to support the findings of this study are available from the corresponding author upon request.
